This article has been retracted.

# The Relationship between Traditional Music in Xinjiang and the Geographical Environment of the Gobi Desert

**DOI:** 10.1155/2022/5610363

**Published:** 2022-07-31

**Authors:** Shuhao Ma

**Affiliations:** South-Central Minzu University, Wuhan 430074, Hubei, China

## Abstract

The natural environment and geographical environment provide the possibility for human survival and development and are also the premise of the formation of music culture. When studying the style characteristics and cultural types of music, more comprehensive and correct conclusions can be drawn only when considering various regional factors such as geography and topographic environment. If we want to explore the music of Xinjiang, we must understand the regional culture. The special geographical location of the Silk Road gives Xinjiang a foreign style compatible with Chinese and Western cultures. At the same time, because of the geographical environment of the Gobi Desert, the music style of Xinjiang is unique. This paper explores the relationship between the traditional music of Xinjiang and the Gobi desert, through the investigation and study of Xinjiang and various musical styles, which have certain reference significance for the study of the Chinese traditional culture.

## 1. Introduction

The formation and development of any national culture must rely on a specific spatial range, but each spatial range is not consistent. As a result of the influence, the resulting national cultural forms are also quite different. As an indispensable part of national culture, music culture runs through ancient and modern times and brings important significance to people's daily lives. When studying the style characteristics and cultural types of music, only by comprehensively considering various regional factors such as geography, landform environment and so on [1] can a more comprehensive and correct conclusion be drawn. China's land area is vast, covering almost all types of landforms such as hills, plains, plateaus, and mountains [2]. Different ethnic groups live in different geographical environments. Each ethnic group speaks different languages and receives different cultural education. This has formed a variety of life and labor patterns, shaped a unique national character and temperament, and created a large number of characteristic musical works [3]. Therefore, if we want to explore Xinjiang's music, we must understand the regional culture [4]. Xinjiang's geographical location is in the center of Eurasia, and many “Silk Roads” pass through the middle, becoming the core of the fusion of Chinese and Western cultures and economies. As the process of cultural and economic exchanges between different regions develops in depth and breadth, the importance of Xinjiang as an open-world platform is even more prominent. The excellent civilizations of ancient India, Babylon, and ancient Egypt collided here, which promoted the final formation of Xinjiang's characteristic regional culture [5]. Xinjiang is located in an extremely arid desert area in the middle temperate zone, with high temperatures and little rainfall throughout the year, surrounded by high mountains, far from the ocean, and closed to the natural geographical environment. However, the more blocked the traffic and the fewer foreign exchanges, the more distinct the regional characteristics will be, and the more complete the local music varieties and styles will be stored [6]. The details are shown in Figure 1. It has historically been at the heart of the political, economic, and cultural intersection of East and West. The four major systems of ancient Chinese culture, Indian culture, Persian culture, Greek culture, and Islamic culture converged here through the Silk Road and influenced each other. Absorb nutrients from it, and on this basis, carry forward the unique regional culture of the nation and pass it on with the development of history. It is also the province with the largest number of neighbours and the longest borders. The national border stretches for several kilometers and accounts for about the total length of our land border. Xinjiang music is best known for Uyghur folk music. It inherits the ancient artistic traditions of Guizile, Gaochangle, Yizhoule, Shule, and Khotanese and retains a strong national character. Due to the geographical separation, in the long-term historical development, Uyghur folk music in various parts of Xinjiang has been infused with the milk of local life, forming several musical color zones with very different styles, namely the southern Xinjiang color area, the eastern Xinjiang color area, and the Daolang color area.

The above-mentioned content of Xinjiang's regional culture restricts the choice of Xinjiang's music themes and styles; the development of Xinjiang's music also promotes the spread of regional culture; and the two influence each other and form a symbiotic relationship. The people of Xinjiang can sing and dance well, so they have the reputation of being “the hometown of singing and dancing” [7].

The various notes and rhythms of music can make us express our feelings of joy or sorrow. The specific geographical environment and the natural environment provide the possibility for the survival and development of human beings and are the prerequisite for the formation of music cultural geography. I have already talked about the way in which the regionality and time and space of the geographical environment act on the music culture and the influence of the geographical environment on the genre and style of music. Xinjiang is a multiethnic area. Xinjiang's folk music has obvious “regional characteristics” in melody and rhythm. The folk music in Xinjiang is mainly dance music, and different regions produce different folk dance music themes. Xinjiang's folk dance can be said to be the treasure house of Xinjiang's music culture, providing many types of music creation materials. Since the piano piece “Three Pieces of Kazakh Dances” created by the people's musician Xian Xinghai based on Kazakh music materials in the 1990s, Chinese composers have used composition theory and composition techniques, combined with the music materials of many ethnic groups in Xinjiang to create a large number of piano works.

## 2. The Influence of Xinjiang's Geographical Environment on Music Culture

The geographical environment of Xinjiang has had a profound impact on the living habits of the local people, and culture with local ethnic characteristics has emerged, resulting in distinctive ethnic traditional music, as shown in Figure 2.

### 2.1. Geography and Landforms of Xinjiang

The overall pattern of Xinjiang can be summarized as “three mountains and two basins”: the northern part of the territory is the Altai Mountains, the southern part is the Kunlun Mountains, and the Tianshan Mountains traverse the middle, and together with the northern Junggar Basin and the southern Tarim Basin, they form the geomorphological pattern of Xinjiang [8]. Xinjiang has a vast territory, surrounded by mountains, far from the sea, and deep inland. Due to the blocking of the mountains, the moist airflow of the ocean cannot reach, so the climate is dry and hot, belonging to the arid and semiarid zone, forming a large desert, and the natural oasis distribution area is small. Xinjiang has the longest inland river in China: the Tarim River. The Tarim River is a kilometer long and is an important river channel in Xinjiang. It is formed by melting icebergs and snow. Xinjiang has the largest desert in China: the Taklimakan Desert. It is a mobile desert formed by the movement of dunes under the action of wind. The area is second only to the Sahara Desert in Africa, ranking second in the world. Xinjiang also has the largest basin in China: the Tarim Basin, which is located between the Tianshan, Altun Mountains, and Kunqi Mountains. Xinjiang is arid and less rainy, with very little precipitation every year, and precipitation is unevenly distributed throughout the region. Xinjiang has a long sunshine time, and the sunshine time is long throughout the year. Because of the sufficient photosynthesis, Xinjiang's melons and fruits are particularly juicy and sweet. However, there is a huge temperature contrast between day and night in most areas of Xinjiang [9]. There are also obvious temperature differences between spring and summer in Xinjiang. In the coldest month, the average temperature in the Junggar Basin is as low as minus degrees. Among them, Fuyun County once became one of the coldest areas in China with a rare low temperature of minus degrees. The hottest place, Turpan, is named “Huozhou” and has become the hottest area in China with high temperatures. The natural environment in Xinjiang is relatively harsh, with a hot and dry climate, large daily temperature difference, and frequent dust and storms. But it is under these living conditions that the willpower of the Xinjiang people to fight stubbornly has been formed. In a tough environment, music has become a great way to treat their pain and depression. Singing, dancing, and poetry from life have naturally become their spiritual sustenance. They are good at dancing. They dance in a simple and unrestrained style and have a typical nomadic temperament. The lofty melody in their singing also reflects their optimistic and open-minded spiritual quality [10].

### 2.2. Unique “Oasis Culture”

“Oasis” refers to a unique production method that exists in Xinjiang. River basins and the surrounding areas of basins are where oases are concentrated, and water sources have become the first consideration for people to migrate and settle. For example, the Hami Oasis, the Hotan Oasis, and the Yanshi Oasis are all based on farming. In the earliest days, oases in Xinjiang were only scattered in large and small river areas, forming a pattern of scattered villages [11]. After passing through Gansu Province, crossed the southeastern part of Xinjiang, and extended eastward to the west coast of Central Asia and North Africa, forming a line that traverses east and west. Due to the severe physical and geographical environmental restrictions, Xinjiang is arid and rainy all year round, surrounded by deserts and sandstorms, and surrounded by large tracts of Gobi and mountains [12]. The spatial index of Xinjiang is shown in Figure 3.

Under this circumstance, the development of agriculture, animal husbandry, and handicraft industry in the oasis area has been affected to a certain extent, but it has brought new opportunities for business development. First, the caravan economy of the Oasis Silk Road has promoted the transformation of the caravanserai into an oasis city-state with the nature of an economic and cultural center, and the economic prosperity has promoted the development of the music culture of the city-states on the Oasis Silk Road. Second, the princes, nobles, and merchants of the oasis city-state, in order to meet the needs of economic and social exchanges, summoned some outstanding folk artists into the princes' or private residences, making them professional artists and then becoming representatives of promoting the development of local music. At the same time, local folk music has also been systematically sorted out, standardized, and improved. Third, the Oasis Silk Road not only promotes the communication of music culture between oasis city-states but also becomes a channel for music exchanges in foreign countries. Fourth, the high development of commerce and handicrafts on the Oasis Silk Road has provided sufficient strength for the advent and development of a variety of musical instruments. Fifth, because religious etiquette is an important carrier of musical activities, the spread of various religions through the Oasis Silk Road in history has had a profound impact on oasis music culture. With the considerable profits brought by commercial trade, not only the villages in the oasis are more prosperous, but also the exchange process between the east and the west is accelerated, which provides the soil for the development of the oasis music culture. Xinjiang's “oasis culture” represents a characteristic of compatibility between Eastern and Western cultures [13]. The special geographical location that there is less communication with the outside world and a large number of local characteristics of Xinjiang are relatively preserved, which provides an opportunity for the formation of national culture. It has become a window for the introduction of cultures from ancient Rome, ancient Greece, ancient India, and other countries. Under the continuous impact of Chinese and Western cultures, Xinjiang Oasis Culture has also continuously absorbed foreign elements to expand the compatibility of its own culture. The ontological characteristics of Xinjiang oasis culture are traditional farming culture, grassland nomadic culture, and various religious cultures [14]. Together with foreign and heterogeneous cultures, a cultural circle of coprosperity has finally been formed, in which various cultures bloom, penetrate, and influence each other. On the premise of keeping its characteristics unchanged, the oasis farming culture has widely embraced other foreign cultures with different attitudes and has integrated various elements into one, which has laid the strong national foundation of Xinjiang oasis culture. In the long-term evolution of history, the oasis culture has also gone through the stage of development-absorption-redevelopment. The Xinjiang nation has developed to the current stage and has actually become the result of the integration of multiple cultures [15]. Whether it is the ancient Silk Road civilization or the current modern civilization, the Xinjiang oasis farming culture has formed unique cultural characteristics after changes and has a long history. Oasis culture is unique, not only in the ecological environment but also in the national character. The culture of a nation is limited by regions, and its economic culture, geographical environment, and historical development trajectory will be different, and people living in this region will also be affected by different cultural existence states in behavior, psychology, and personality [16]. Xinjiang oasis culture embodies integration, diversity, and integration. Therefore, it is not only the product of the role of the purely regional environment but also the result of the coexistence of oasis characteristics and heterogeneous cultures. Most of the cultural forms of oasis music represent the real life of local people and also include various cultural elements such as local legends, literati poems, and philosophical words [17]. We investigated and analyzed the learning situation of long and short tones, and the specific results are shown in Figure 4. The results found that the majority of the traditional Mongolian songs were vague.

## 3. The Basic Introduction of Xinjiang Folk Music

### 3.1. The Historical Origin of the Formation of New Style Music

Xinjiang is located in the central region of Central Asia, which is of great significance in connecting the East and the West and promoting regional economic and cultural development. The longest section of the Silk Road is located in Xinjiang, China (Table 1). This section of the commercial road is more than 2,000 kilometers long and is a very important transportation hub on the “Silk Road.” The essence of ancient Chinese culture, Indian culture, Greek culture, and Islamic culture is integrated here, and based on this, a characteristic regional culture with Xinjiang style has been formed [18]. The melody of Xinjiang folk music is beautiful; the rhythm is lively and distinct; the structure is regular and symmetrical; the mood is warm and cheerful; most of them adopt the seven-tone natural mode; and there are also five-tone modes: b7, #1, #2, #4, and #5; and the main accompaniment instruments are tambourine, dongbula, rewafu, iron drum, and so on. The lyrics are easy to understand, and Uyghur's famous large-scale national music and dance epic “Twelve Mu Kam” has long been circulated among the people and is deeply loved by the masses. Going back to the origin of music, Xinjiang is mainly influenced by three major systems: Mongolian system, Iranian music system, and European music system. The main characteristics of these three music systems can be summarized as shown in Table 1.

Generally speaking, the typical music style of a region is usually represented by the folk songs of the region because folk songs are the crystallization of the unique society and human culture of the region after years of development and evolution and then processed by people [19]. Xinjiang has always been a multiethnic area in history, and among the thirteen ethnic groups living in it, Uyghur, Han, Kazakh, Kirgiz, and Tajik are the most representative. Because these five ethnic groups have already lived in Xinjiang before Turkicization, it is necessary to study the musical styles of these five ethnic groups in order to understand the historical origins of Xinjiang's musical styles. Du Yaxiong showed in his research results that the formation of a national musical style is closely related to the ethnic characteristics of the ancient ancestors of the nation, rather than the religious beliefs, the inhabited areas of the nation, or the national language. The ancestors of the Han nationality migrated from the Central Plains, and the race belongs to the branch of Mongolia, so the music of the Han nationality reflects the style characteristics of the Mongolian system [20]. The ancestors of the Xinjiang people are mainly the Uighur people, which were renamed from the Ouigour people, and also included the residents from Iran and primitive Europe. These three parts are the main sources of the original residents of Xinjiang, as shown in Figure 4. Mongolian music is characterized by a distinct national style: beautiful melody, wide atmosphere, deep feelings, and strong grassland atmosphere. Mongolian music is dominated by folk songs and raps associated with nomadic life. There are traditional ancient hymns, hymns, feasts, and many songs that reflect the lives of herders. Mongolian folk songs are divided into two types according to their musical characteristics: “Urtu” songs (i.e., long-key songs) and “Uhur” songs (i.e., short-key songs). The former has a free rhythm and a long breath, with a slow speed and a wide range of sounds; the latter has a distinctly regular rhythm and a brisk speed.

Each of these three systems has its own characteristics: Huiya belongs to the Mongolian race. The main features of this type of race are long faces and high cheeks. They migrated from east to west to the Hami area of eastern Xinjiang more than 3,000 years ago; the Iranian race originated from the ancient eastern Mediterranean region; and Pamir-Fergan is a branch of primitive Europeans, and the typical feature of this race is the short face, which first appeared in the Ili River Basin in Xinjiang. The Pamir-Fergan type is closely related to primitive Europeans, so researchers regard this species as the result of the evolution of primitive Europeans. Since the formation process of the Uyghur nation is influenced by the three types of ethnic groups, the music style also has the characteristics of the Mongolian system, the Iranian system, and the European system. Taking the Kazakhs as an example, going back to the historical origin, the formation of this nation comes from two major systems: one is the Pamir-Fergan, which belongs to the primitive Europeans; the other includes the Huiya and Khitan tribes, which belong to Mongolia. Therefore, Kazakh folk music has the common stylistic characteristics of the two systems. The ancestors of the Kirgiz people came from the Lianghe region of Europe and belonged to primitive Europeans. They lived in the southern part of Xinjiang and were the product of the great migration and integration of residents. Therefore, the national music style of the Kirgiz people has the characteristics of the Persian-Arab system and the two European systems. The ancestors of the Tajiks originate from the Xian, which is related to the Mongolian race. Therefore, the music of the Tajiks has the characteristics of the Mongolian system. From the analysis of the musical characteristics of the above-mentioned ethnic groups, we can comprehensively analyze the formation of the musical styles of each ethnic group from the perspective of one or several musical systems to which they belong.

### 3.2. Piano Music Works in Xinjiang Regional Culture

The creation of Chinese piano music is based on the materials of Chinese folk music, and it is significantly different from Western piano music in terms of tonality, harmony, and creative techniques. The earliest Chinese piano music works were adapted from Chinese folk songs, and the music theme adopts the melody widely circulated in folk songs, with obvious Chinese pentatonic color in debugging. China has a vast territory, so Chinese piano music reflects the cultural characteristics of many regions. Every nation and every region has its own unique regional culture. National music takes regional culture as the cradle and breeds musical styles that are different from other regions. As the carrier of music, the piano improves the creation of folk music and enriches Chinese piano works. It uses piano skills to push folk music to a newer and more mature stage so that the music works have distinct regional characteristics. The differences in regional culture have led to different styles of Chinese piano music works, and many places have their own representative piano works. The details are shown in Table 2.

## 4. The Regional Environment of Xinjiang Determines the Characteristics and Content of the Piano Music in Xinjiang

### 4.1. The Characteristics of Xinjiang's Piano Music

Xinjiang plays an important role in connecting the Eurasian continent and has a major strategic position. At the same time, it is also the intersection of ancient Chinese culture in the east, Indian culture in the south, Greek culture in the west, and Islamic culture in the southwest. This sparked a fierce spark and brought sufficient nutrition to the economic and cultural development of Xinjiang. Xinjiang's special geographical location determines its historical status. The terrain of Eurasia is mostly high mountains and dense forests. There are three Silk Roads running through it, all of which pass through Xinjiang. The north road goes around the northern part of the Tianshan Mountains in Xinjiang; the south road passes through the south of the foothills of the Tianshan Mountains in Xinjiang; and the inner and outer routes pass through Kuncang Mountain. These three Silk Roads have brought huge development opportunities to the development of the Xinjiang region, making the Xinjiang region a hub for cultural, artistic, and economic exchanges between countries. Xinjiang Uyghurs have lived on this Silk Road for generations. This superior geographical environment makes it easier for Uyghurs to absorb the essence of Persian, ancient Rome, ancient Greece, and other exotic civilizations for their own use, which is conducive to the widespread use of Uyghur music culture. The Uyghurs, known as the Uighurs, lived in the Mobei region. There are two ancestors of Huihe cranes: one is Dingling, which is an ancient nomadic people living in the area of Lake Baikal, once under the jurisdiction of the Huns. Later, the Huns were defeated by the Turks, and Ding Ling began to embark on the road of independent development. During the Wei, Jin, and Southern and Northern Dynasties, Xinjiang experienced a stage of national integration. The Tubo, Yuezhi, Xian, Rouran, Wusun, Xiongnu, Tubo, Huihe, and so on moved into Xinjiang one after another and lived together with the original residents of the Tarim Basin, forming a multiethnic living pattern. After the Uighurs migrated westward, they were influenced by the Han culture in the Central Plains and the four ancient civilization systems and finally formed the Uyghur nation and Uyghur culture. “Uyghur” means “unity” in the Uighur language. The diverse regional culture makes Xinjiang music inclusive and integrates the elements of folk music from many ethnic groups in Xinjiang, including the three-beat juniper melody and the jumping drum beats. Rhythm. Xinjiang's oasis culture is a regional culture with national characteristics, which endows the people of Xinjiang with a national character of perseverance, which is expressed in the style of music with enthusiasm and liveliness, which is not possessed by ethnic groups in other regions. Xinjiang style piano works have unique artistic charm in melody by using the rhythm combination of round dot, cut, first sixteen, last eight and weak rise. Moreover, they use parabolic melody such as wave, small second and increased second, and other special intervals, “true” and other techniques. The creation of piano works in Xinjiang style shows xinjiang's unique famous scenery and magnificent, vicissitudes of life, and colorful regional scenery. Xinjiang music reflects the influence of regional culture on it, which is reflected in four aspects: beat, rhythm, melody, and harmony as shown in Table 3.

### 4.2. The Content of Xinjiang Piano Music

The characteristics of rhythm, beat, melody, and harmony in the above-mentioned piano works are unique to the Xinjiang region and cannot be seen in the musical works of other regions. Although Xinjiang-style piano works are numerous and vast, because their creations all originated in the same region, they are constrained by similar geographical environments and cultural background and have similarities in the characteristics of the music itself. Therefore, we can understand the specific regional cultural content of Xinjiang ethnic group from several piano works with typical Xinjiang style. Sun Yiqiang's piano work “Spring Dance” and Ding Shande's “Second Xinjiang Dance” mentioned above were written based on the cultural background of the Xinjiang ethnic group. For each musical form, we investigated the popularity of their works among students, as shown in Figure 5. According to the results, most students still prefer pop music, and only 10% of the students like folk music.

First, it reflects the Uyghur people's enthusiastic and eloquent national character, as well as the national custom of being good at dancing. The Uyghurs are one of the main ethnic minorities in Xinjiang. They are best at performing dance types with strong rhythm, prominent drums, multiple rotations, and unrestrained movements. The inspiration for Sun Yiqiang's creation of the piano piece “Spring Dance” came from the hand drums of the Uyghur people in Xinjiang. It was a common dance in sacrificial activities at first. Women were the main body of the dance, and men were accompanied by hand drums. The artist's adaptation and development have become the hand drum we see today. The author draws on the syncopated rhythm of hand drums and the typical musical rhythm in the creation process. The piano piece “Spring Dance” is very brisk in rhythm, with prominent rhythm and accent, which reflects the overall style of Xinjiang dance's free and easy movements and rapid rotation. In addition, the language characteristic of the Uighur language is that the accent is placed on the last syllable of the multisyllable, resulting in iambic, which is also a reason why the syncopated rhythm is widely used in Xinjiang-style piano works.

Second, it reflects the positive and optimistic national temperament of the Xinjiang people. In the introductory part of “Spring Dance,” the author enters in a major key, laying the foundation for the bright colors of the whole song, and the slightly random rhythm has room for free handling, leaving room for people to continue to develop reverie. The use of this kind of loose board also draws on the creation method of Xinjiang's cultural treasure “Twelve Muqam.” “Twelve Muqam” is relatively free in the first paragraph, and there is no fixed requirement for rhythm, so it is relatively free. The loose board in the first half is mainly to pave the way for the development of the later music, resulting in the characteristics of first depression and then rising. The theme melody of “Spring Dance” appears many times. The left-hand part uses a continuous syncopated rhythm to maintain a stable rhythm. The right-hand melody changes and repeats. Continue to move forward.

In addition, most of the piano songs “Spring Dance” adopt upward melodies so that the music continues to develop so that the whole piece presents a warm and positive musical atmosphere. In terms of overall musical style, it maintains the strong ethnic and regional characteristics of the Uyghur people in Xinjiang. The rhythm not only reflects the synchronous rhythm of the tambourine but also highlights the main connotation of the warm and unrestrained drum in the melody of Xinjiang, as well as the excellent tradition of the oasis people's positive national character and not being afraid of difficulties. It has endowed the Xinjiang nation with a tenacious national temperament and an optimistic attitude towards life.

Third, Xinjiang piano music is also reflected in the similarity and compatibility of traditional ethnic instruments in Xinjiang, such as the plucked instruments Dongbula and Rewafu. The expressiveness of the instrument is often used to set off the warm and cheerful rhythm and melody. Dongbula is a common piece of music in Xinjiang. It can be played with a wide range of sounds, bright timbre, and vivid and diverse performance forms. Rewaf is a wooden musical instrument, often used to play brisk and lively tunes. The bass accompaniment part of “Spring Dance” usually highlights the rhythm and accent and is clean and neat, just like playing the traditional musical instruments of the Xinjiang people, which is refreshing.

Fourth, it reflects the cultural characteristics of Xinjiang's inclusiveness. Xinjiang is located in the central region of Central Asia, which is of great significance in connecting the East and the West and promoting regional economic and cultural development. Going back to the origin of music, Xinjiang is mainly influenced by the Chinese music system, the Persian-Arabic music system, and the European music system. Therefore, the folk music of the Xinjiang ethnic group has the characteristics of these three systems. Natural minor, harmonic minor, mixed Lydian, and Dorian are the most commonly used modes in European music systems. Ding Shande's “Second Xinjiang Dance” uses the Dorian mode in the European music system, and the main tone is the tone. This ancient European mode presents a new look in the process of combining with the traditional mode of Xinjiang folk music and has been further inherited.

The piano pieces “Spring Dance” and “Second Xinjiang Dance” occupy an irreplaceable position in the history of Chinese piano music with their respective artistic charms, showing the strong “regional flavor” of Xinjiang. By imitating hand drums, it shows the dynamics of drum beats and reflects the humor of Xinjiang people in the vast Gobi desert and the oasis with lush water and grass; it conveys from the tune that Xinjiang is vast and sparsely populated, and the harsh living environment determines Xinjiang. People must rely on each other and help each other to survive the heroic, magnificent, and helpful regional characteristics; from the mood of the work, it shows the prosperity brought by the Silk Road and the colorful regional cultural characteristics of the fusion of Chinese and Western cultures.

## 5. Conclusion

Musical culture has a direct origin in human life and production activities and methods, and regional differences affect this way of life. For people living in the same area, the natural environment is the same, and the ideas derived from the ideas acting on the human heart are also similar. From another perspective, aesthetic concepts and personality traits in turn prompt people to make different choices about their environment. Therefore, the musical cultural events bred by the above factors have typical regional differences. There is a strong link between regional culture and music. The production and development of music are based on the time and space of a certain region, reflecting the cultural characteristics of the region.

Xinjiang has a long regional history, has a unique geographical location, plays an important role, and has experienced multiparty integration in cultural development, and under the joint action of these factors, a characteristic regional culture with Xinjiang style has been formed. Oasis culture is a cultural orientation that Xinjiang people have always admired, and it is also a characteristic product of Xinjiang's regional culture. It represents the optimistic ideology and spiritual outlook of the Xinjiang nation. This humanistic culture has created a strong sense of rhythm and dance style in Xinjiang music. From the perspective of these musical works regionally, it is not difficult to find that the piano works in the Xinjiang genre and style have significant regional characteristics in terms of rhythm, rotation, rhythm, and other musical ontology, which is unique in Xinjiang. Regional culture is the soil for the production of musical works, providing a material basis for music creation. Music can promote the development of regional culture, and with music as the carrier, regional culture can be promoted. As a result, there is a coexistence between regional cultures and music, interdependent. The long history and culture have created a splendid civilization in Xinjiang. The special geography of the Silk Roads gave Xinjiang an exotic atmosphere compatible with Chinese and Western cultures. It occupies an important position in the creation of Chinese piano music and is loved by more and more people.

## Figures and Tables

**Figure 1:** The relationship between traditional music in Xinjiang and the geographical environment of the Gobi Desert.

**Figure 2:** The influence of Xinjiang's geographical environment on music.

**Figure 3:** Spatial pattern index of Xinjiang folk music.

**Figure 4:** Statistical chart of student learning results.

**Figure 5:** Students' love for all kinds of music.

**Table 1:** Main characteristics of the three music systems.

	Mongolian system	Iranian system	European system
Tone structure	Tone with cavity	Tone conditionally with cavity	Tone without cavity

Music organization	1. The mode is based on three tones and four groups	1. The mode is based on the four-tone series	1. The mode is based on the four-tone series
	2. Pentatonicity of tones	2. Melody has no functional and surface meaning	2. Melody has functional and surface meaning

Beat rhythm	1. Loose plate	1. There is a board (characterized by a fixed rhythm pattern)	Rhythm with a board
	2. Nonrhythmic board	2. Loose plate	
	3. The rhythm has a board	3. Mix the beats	

Texture characteristics	Mainly lateral thinking	Lateral thinking, but when there is a fixed rhythm pattern IV, it shows the characteristics of vertical thinking	Mainly vertical thinking

**Table 2:** Regional characteristics of each region and representative works of piano music.

Area	Representative work
The Loess plateau is located in the northern Shaanxi region of China. The natural environment there is harsh, stormy weather, road asaki woman, but living in the area of people cheerful and optimistic, not afraid of real harsh conditions, create a style of coarse mining atmosphere piano works	Its representative works are Wang Jianzhong's “Shan Dan Dan Blossom Red” and Zhou Guangren's “theme variations of North Shaanxi folk songs.” The theme of “Shan Dan Dan Blossom Red” is based on the traditional folk song “when the red army brother comes back” in northern Shaanxi. It depicts the welcome scene of the people in northern Shaanxi when the red army returns from winning the battle. The music is cheerful and clear and beaming.
The nomads of the Inner Mongolian grasslands love the blue sky and white clouds, the galloping eagles, the endless grasslands and the unrestrained freedom of life. Inner Mongolia people treat the distant guests sincerely, with warm and straightforward character, so the Mongolian music style is simple and moving, with melodious melody, straight through the people's hearts.	His representative work is “seven theme songs of inner Mongolia folk songs” by Sang Tong. The seven songs include “memorial,” “friendship,” “homesickness,” “prairie love song,” “the children's dance,” “grief,” and “dance”; the piano works are in inner Mongolia local folk songs, for its melody, rhythm, and the content of the music to reflect the daily life of inner Mongolia people.
Guangdong area is located in the south of China, with a superior geographical environment and a comfortable and pleasant climate. Therefore, the Guangdong music tune is light, compact rhythm, delicate and small structure, with elegant and chic-style characteristics.	Guangdong area is located in the south of China, with a superior geographical environment and a comfortable and pleasant climate. Therefore, the Guangdong music tune is light, compact rhythm, delicate and small structure, with elegant and chic-style characteristics.
Yunnan-Guizhou Plateau area is mostly mountainous; influenced by its specific geographical environment, the music works of Yunnan-Guizhou area usually have a strong folk song characteristics; and the melody line is broad and long, easy to be sung between the mountains of qi women. Most of the music in this area adopts the way of flat and straightforward narration, with less decoration and relatively simple structure.	His representative work is zhu Jian's running water, which is a reflection of the simple life of people living in the area. Sichuan is located around the Qinghai-Tibet plateau, with numerous ethnic minorities.
Music in Sichuan area is obviously affected by its geographical environment, and the high mountains are the natural barrier to nature. People living in this region love nature and advocate a simple way of life, so they form a relatively free and casual music style, and have no fixed rhythm mode.	People living in Sichuan love nature and advocate a simple life style, so the music they like is a free and casual style without a fixed rhythm pattern.

**Table 3:** The beats, rhythm, melodies, and harmonies of Xinjiang music.

Meter	Mix beats, change beats, and loose plate beats
Rhythm	Weak rhythm, attached point rhythm, syncopated rhythm, triple link rhythm
Melody	Parabola type, top true type, song head type
Harmony	High stack processing of the chord, pentatonic chords, sound structure, compound chord, parallel harmonic progress, stubborn progress

## Data Availability

The labeled data set used to support the findings of this study is available from the corresponding author upon request.
